This article has been retracted.

# Software Application toward Accessible Hearing Care Assessment: Gap in Noise Test

**DOI:** 10.1155/2022/1112598

**Published:** 2022-04-29

**Authors:** Khalid Alhussaini, Shaza Saleh, Adham Aleid, Saad Alkhalaf, Reem Badghaish, Amir Altinawi, Abdullatif Alwasel

**Affiliations:** ^1^Department of Biomedical Technology, College of Applied Medical Sciences, King Saud University, 10219 Riyadh, Saudi Arabia; ^2^King Abdullah Ear Specialist Center, King Abdulaziz University, King Saud University, 10219 Riyadh, Saudi Arabia; ^3^Ear Institute, University College London, London, UK

## Abstract

Currently, several methods are being applied to assess auditory temporal resolution in a controlled clinical environment via the measurements of gap detection thresholds (GDTs). However, these methods face two issues: the relatively long time required to perform the gap detection test in such settings and the potential of inaccessibility to such facilities. This article proposes a fast, affordable, and reliable application-based method for the determination of GDT either inside or outside the soundproof booth. The proposed test and the acoustic stimuli were both developed using the MATLAB® programming platform. GDT is determined when the subject is able to distinguish the shortest silent gap inserted randomly in one of two segments of white noise. GDTs were obtained from 42 normal-hearing subjects inside and outside the soundproof booth. The results of this study indicated that average GDTs measured inside the booth (5.12 ± 1.02 ms) and outside (4.78 ± 1.16 ms) were not significantly different. The measured GDTs were also comparable to that reported in the literature. In addition, the GDT screening time of the proposed method was approximately 5 minutes, a screening time that is much less than that reported by the literature. Data show that the proposed application was fast and reliable to screen GDT compared to the standard method currently used in clinical settings.

## 1. Introduction

The World Health Organization (WHO) estimates that around 2.5 billion people will experience hearing impairments by 2050 [1]. Therefore, the need for hearing care services is growing worldwide in both developing and developed countries. However, developing countries are more susceptible to poor accessibility to hearing care services due to financial means and logistical challenges. Moreover, one of the solutions for healthcare accessibility is implementing telemedicine or self-administered medical diagnostic tests. Generally, there is significant room for improvement in hearing assessment by utilizing self-administered screening tests.

Furthermore, hearing care may not be affordable in first-world countries due to fact that some medical insurance plans may provide inadequate or limited coverage for hearing care [2, 3]. In addition, large populations in the low economic countries may not have accessibility to hearing care services due to the financial inability of their health sectors to establish audiology clinics, which require medical devices, furniture, construction, and other overhead costs [4–7]. An affordable and accessible alternative to tackle these concerns is using the available technology in smartphones and low-cost sensors [8, 9].

Several medical diagnostic purposes have witnessed the development of affordable and accessible point-of-care (POC) testing, which refers to the fast acquisition of certain patient clinical information at the desired time outside the conventional laboratory settings. POC reduces turn-around time, which is the time taken from test requests to test results, provides early detection, and reduces the need for human and technical resources [10, 11].

In audiology, developing affordable and accessible technologies for hearing would allow early detection of hearing abnormalities, reduce the cost of the medical systems, and increase the accessibility of hearing care to all patients in need. However, to rely on self-administered tests in hearing screening/evaluation, a validation process should be performed to ensure comparable effectiveness and accuracy as traditional tests performed in clinics. Several hearing tests outside the clinical setup have shown significant validity [12–15]. For example, Na et al. [16] developed a smartphone hearing screening application to be used in a noisy environment. By utilizing built-in microphones in smartphones to measure the noise level and correct the audiogram values, they improved the test values to match those values obtained in a clinical setup [16].

Although many affordable, self-administered hearing screening tests have been proposed and validated, the audiology testing battery performed in the clinic is not limited to obtaining audiograms. Speech in noise test, gap in noise test, and sound source localization test are examples of the behavioral tests performed to assess specific skills in hearing and speech perception. In particular, the gap in noise test is a commonly applied test protocol in the clinical setting to evaluate and diagnose the status of auditory temporal resolution. The test reflects the shortest silent gap duration perceived by the human ear [17–19]. Auditory temporal resolution is a measure of gap detection threshold (GDT), in which the elevation from the normal value of about 5 ms may indicate an abnormality [17]. Although temporal resolution is one of the components of auditory processes, neurological disorders often accompany anomalies in auditory processing. Disorders such as autism, multiple sclerosis, and auditory neuropathy are common examples [20]. Additionally, older adults are prone to degraded temporal resolution as they get older [20]. Moreover, normal speech perception correlates with intact temporal processes [21, 22]. Therefore, the need for accessible, easy to administer temporal resolution assessment tests is deemed essential to evaluate and diagnose such conditions.

This study explores the feasibility of self-administered, computer-based tests to assess temporal resolution by obtaining GDTs. For validation purposes, GDTs are obtained under two different settings (inside and outside a soundproof booth). This protocol permits investigating the reliability of the computer-based application in determining GDT in circumstances that lack the traditional clinical setting.

## 2. Methods

Experiments of measuring GDT levels, using the proposed user interface application, were performed on all 42 male and female participants inside and outside the soundproof booth. Experimental data were collected and statistically analysed in order to investigate the influence of ambient noise on the determination of GDT level, hence validating the use of the proposed user interface application outside the soundproof booth.

### 2.1. Participants

Twenty-one female and twenty-one male subjects with normal-hearing levels volunteered in this study. All subjects participated in both the “IN-test” (i.e., measuring GDT inside the soundproof booth) and the “OUT-test” (i.e., measuring GDT outside the soundproof booth). The age of the participants ranged from 20 to 43 years with a mean of 27.8 ± 6.5 SD years. The hearing threshold of all subjects was 30 dB HL or better for the 250 to 8000 Hz octave frequencies. The study was approved by Institutional Review Board (IRB) at the College of Applied Medical Sciences, King Saud University (CAMS 029-3940). Written consent to participate in the study was signed and obtained from all participants in the study.

### 2.2. Stimuli

During the OUT-test, all participants were tested outside the soundproof booth in which the ambient noise existed. Before each test, the ambient noise level was measured using a sound level meter (Extech 407730: Digital Sound Level Meter). Ambient noise intensity during the OUT-test ranged from 45 to 50 dB. On the other hand, all participants were tested in a controlled environment inside the soundproof booth throughout the IN-test. In each IN-test and the OUT-test trial, participants listened to two acoustic stimuli segments using headphones set (Sennheiser HD 280 Pro) that was previously investigated and proved acceptable for audiometry screening [23, 24]. The noise segment characteristics and silent gap envelope design were described and applied in previous studies [25, 26].

A silent gap randomly appeared in one of the two 1 sec duration acoustic segments. To minimize the prediction memory-based effect [27], the silent gap location within the segment was varied randomly in each trial. A 10 ms slope characterizes the acoustic stimuli waveform at the white noise segment's beginning and end. The slope of the silent gap inserted in the noise segment was 1 ms to avoid sudden abrupt change from sound to silence, which may lead to a click effect.  Figure 1 shows a schematic illustration of the experimental setup, stimuli signals and slopes, and user interface window.

The subject receives the stimuli (with and without gap) through the headphones and responds by pressing either “1,” “2,” or “I DON'T KNOW” button to indicate hearing the gap in the first segment, in the 2-sec segment, or uncertainty about hearing the silent gap, respectively.

### 2.3. Software Setup

The user interface and the acoustic stimuli of the computer-based application were both developed using MATLAB®. As mentioned above, the gap detection test contained a series of testing trials, each of which comprises two acoustic segments of white noise with a silent gap inserted randomly in one of the two segments. The silent gap durations presented ranged from 20 ms down to 2 ms.  Figure 2 illustrates how the test is acquired in a relatively short period by focusing on tuning around expected thresholds. As shown in Figure 2, the large step size reduction in the gap duration in phase A determines a 4 ms threshold region (GS_region_). Each GDT is detected and saved during phase B. Whenever the algorithm registers a larger number of false responses (FSs) compared to that of the positive responses (PSs), phase A is terminated, and the threshold region (GS_region_) is registered. At this point, phase B is initiated with a small step size decrease (1 ms) in the gap duration for fine-tuning and determination of expected GDT within the specified GS_region_, also when the number of FS is larger than that of PS.

Phase A is used to determine the threshold region (out of 4 threshold regions: 20-16, 16-12, 12-8, and 8-2 ms). Phase B is the fine-tuning and GDT determination phase within the specified threshold region. GS: gap size; PS: positive response; FS: false response; GDT: gap detection threshold.

The application user interface window contained three buttons. The two buttons are labeled “1” and “2” referring to the selection of first and second stimulus segments, respectively, whereas the button labeled “I DON'T KNOW” refers to the uncertainty about hearing the silent gap.

### 2.4. Data Collection

In the beginning, subjects were informed about the purpose and details of the experiment. Then, each participant signed the informed consent. Prior to the GDT evaluation, each subject was administered a conventional pure-tone behavioral hearing test using a clinical-grade audiometer. All subjects included in the study showed normal hearing (with thresholds ≤30dBHL at 0.25, 0.5, 1, 2, 4, and 8 kHz) and reported no neurological disorders.

Then, participants were randomly divided into two subgroups. The first group included 21 subjects (11 females and 10 males), whereas the second group included 21 subjects (10 females and 11 males). All participants performed both the IN-test and OUT-test in a random order according to the group. Participants in the first group completed the OUT-test first and then the IN-test, whereas subjects in the second group performed the reverse order (IN-test first and then the OUT-test).

In each test, the subject was instructed to use the application user interface window to press button “1” or “2” to select the acoustic segment having the silent gap or to press the button “I DON'T KNOW” if he/she was not sure about hearing the gap. In addition, participants had the chance to practice the task before the actual test to ensure that they got used to the system.

## 3. Results

Each participant performed the gap detection test twice: OUT-test and IN-test. While the first group carried out the OUT-test first, the second group carried out the IN-test first.  Figure 3 shows GDTs (mean ± SD) of all 42 participants obtained from the IN-test (5.12 ± 1.02 ms) and the OUT-test (4.78 ± 1.16 ms), regardless of the test order or participant gender.

GraphPad Prism version 9.1.2 was used to carry out statistical analysis. Nonparametric tests were applied since Shapiro–Wilk's test revealed that the GDTs of the OUT-test condition, the IN-test condition, males, and females were not normally distributed. Wilcoxon signed test showed that there was no statistically significant difference in the GDTs between the results of the OUT-test condition and that of the IN-test condition for the whole group (*Z* = −112, *N* = 42, *p* = 0.1) or for the female group (*Z* = −28, *N* = 21, *p* = 0.19) or for the male group (*Z* = −31, *N* = 21, *p* = 0.35).

42 subjects performed both the OUT-test and IN-test. There is no significant difference between the results of the two tests.

Figure 4 shows the GDTs for the two groups, taking into account test order (either starting with the IN-test first or starting with the OUT-test first). There was no statistically significant difference in values of GDTs obtained from the IN-test between the two groups, nor in the values of GDTs obtained from the OUT-test between the two groups (*p* value = 0.16, ANOVA test).

There are 2 sets of participants (each set includes 21 subjects) who performed both the IN-test and OUT-test in a different order. The first set started with the OUT-test (black), whereas the second set started with the IN-test (gray). There is no significant difference among the GDTs of any of the four data sets.

Figure 5 shows the GDTs for the same two groups classified according to gender and test type (IN or OUT) regardless of which test was performed first. Mann–Whitney test revealed no statistically significant difference in the GDTs obtained from males and females for the IN-test (*U* = 202, *p* = 0.63) nor the OUT-test (*U* = 202, *p* = 0.96). Likewise, Wilcoxon signed test showed no statistically significant difference in the values of GDTs obtained from the OUT-test whether it was applied as the 1st or the 2nd condition (*Z* = −45, *N* = 21, *p* = 0.12) nor in the values of GDTs obtained from the IN-test (*Z* = −55, *N* = 21, *p* = 0.16). This result suggests that there was no order (IN-test vs. OUT-test) effect.

There are 21 male participants (in black) and 21 female participants (in gray) who all performed both the IN-tests and OUT-tests. There is no significant difference among any of the four data sets.

Values of GDT (mean ± SD) for 21 male participants (in black) and 21 female participants (in gray) who all performed both the IN-test and OUT-test. There is no significant difference among any of the four data sets.

## 4. Discussion

The gap in noise test is currently performed in a clinically controlled setup using a soundproof booth [17, 19]. With the different socioeconomic and geographical constraints that could impede patients' access to this essential auditory screening, there was a need to develop and test a reliable method to determine the GDT outside the clinical environment. Most recently, Alhussaini et al. [23] introduced a computer-based application for GDT evaluation. This study applied this method to normal-hearing adults (age range of 20–43) to investigate its suitability to evaluate auditory temporal resolution. In 2000, a consensus of experts recommended that a gap in sound tests should be used to assess auditory temporal processes [28].

The results of the current study indicate that, regardless of gender, there was no significant difference in the GDT measured levels whether the measurement was carried out inside the soundproof booth or outside the booth with ambient background noise in the 45–50 dB range. In addition, adopting the idea of threshold region (phase A) in the proposed test had a great contribution in shortening the time required to acquire GDT down to about 5 minutes. This GDT acquisition time is much lower than that of the commercially available GIN test, which takes about 17 minutes to acquire GDT [17].

Applying the proposed gap detection test remotely to different populations, for instance, cochlear implant (CI) recipients or hearing aid (HA) users, can further enhance teleaudiology by incorporating it to evaluate outcomes or guide change in settings. In addition, evaluation of ease of use in these populations and establishing normative data for them with this application could significantly push forward the application of this test remotely and utilize its results in the remote fitting of CIs and HAs.

Additionally, the proposed test can be applied remotely to target school-aged children in their educational settings without specialized equipment or costly soundproof booths. This test can detect temporal auditory issues that may lead to low school performance [29] or specific language disorders [30, 31], particularly if undiagnosed.

The proposed application can be a valuable tool for the early detection of possible auditory temporal resolution problems in younger children by making it a child-friendly and self-rewarding application. Such an approach may allow for early intervention and contribute to reducing language development problems related to auditory temporal resolution problems. Within the same context, the application may be used remotely in preschools as a screening test.

## 5. Conclusions

The proposed application-based method produced comparable thresholds whether administered inside or outside the soundproof booth. The results of this method demonstrated fast, affordable, and reliable GDT screening with the lack of a controlled clinical setting.

However, the presented findings need additional validation by applying the same procedure to hearing-impaired patients and to a broader age span to cover older adults who are known to develop lower GDT in comparison to normal hearing adults. Moreover, establishing normative data for different populations (e.g., young children and cochlear implanted patients) could expand the use of the proposed application-based method. This method was a step toward developing a reliable remote software-based screening tool that makes these services available in rural areas and underdeveloped countries.

## Figures and Tables

**Figure 1:** The experimental setup includes stimuli, participant, headphones, and user-interface window.

**Figure 2:** Summarized representation of gap detection software algorithm flowchart.

**Figure 3:** GDTs (mean ± SD) from the OUT-test and IN-test.

**Figure 4:** GDTs (mean ± SD) from the OUT-test and IN-test performed in a different order.

**Figure 5:** GDTs (mean ± SD) from the OUT-test and IN-test classified with respect to gender.

## Data Availability

The data used to support the findings of this study are available from the author upon request.
